# PTPN11 Gene Mutations and Its Association with the Risk of Congenital Heart Disease

This article has been retracted.

**DOI:** 10.1155/2022/8290779

**Published:** 2022-04-09

**Authors:** Zi-qing Xu, Wei-cheng Chen, Yu-jie Li, Mei-jiao Suo, Gui-xiang Tian, Wei Sheng, Guo-ying Huang

**Affiliations:** ^1^Children's Hospital of Fudan University, Shanghai, China; ^2^Shanghai Key Laboratory of Birth Defects, Shanghai, China

## Abstract

Congenital heart disease (CHD) is the most common congenital birth defect, with a prevalence of 8.98‰ of all live births in China. PTPN11 has been known to be closely involved in heart developments. In this research, we carried out whole-exome sequencing in nine CHD families and identified eight rare deleterious missense variants of PTPN11 gene in nine probands by stringently filtering criteria. Sanger sequencing of these probands and their unaffected familiar members revealed that six damaging variants were de novo in seven CHD families. Then, targeted sequencing was used to assess the PTPN11 exon variants in 672 sporadic CHD cases and 399 unrelated controls and identified 7 deleterious missense variants in 8 patients. Fisher's exact test reveals a significant association of PTPN11 variations with CHD (*P* = 0.0289). We observed the distribution of different subtypes in CHD patients with PTPN11 variants and found atrial septal defect (ASD) is a prominent phenotype (58.8%, 10/17). In vitro functional assays revealed that the predicted PTPN11 variants disturb RAS-mitogen-activated protein kinase signaling activity by influencing the phosphorylation level of pathway proteins and increasing the proliferation and migration abilities of cardiomyocytes to different extents. Our findings demonstrated that PTPN11 variants were associated with increased risk of CHD development and may be served as an important susceptible genetic event for CHD, especially the ASD subphenotype.

## 1. Introduction

Congenital heart disease (CHD) is a cardiovascular formation or developmental disorder that occurs during embryonic development. It is the most common congenital birth defect, with a prevalence of 8.98‰ of all live births in China [1]. CHD etiology is multifactorial, involving genetic and environmental components [2]. An estimated 400 genes are implicated in the pathophysiology of CHD, including transcription factors, cell signaling molecules, chromatin modifiers, and structural proteins essential to heart developments [3, 4]. The specification, differentiation, and patterning of heart cells can be hampered by mutations in these genes, resulting in changes to the heart's structure and function.

Previous studies have confirmed the correlation between PTPN11 gene function and heart development in various animal models such as mice [5–7], zebrafish [8–10], and Xenopus [11, 12]. In fact, PTPN11 is closely related to important biological processes including cardiac progenitor cell differentiation [11], cardiac circularization [12], endocardial cushion and valve development [13–15], and maturation and separation of the heart cavity [5].

PTPN11 gene encodes the protein tyrosine phosphatase (PTP) SHP2, which is an important member of the PTP family that works with phosphokinase to maintain the homeostasis of the whole internal environment. SHP2 contains three main functional domains, including two tandemly arranged SH2 domains at its N-terminal end (N-SH2 and C-SH2) and a catalytically active PTP domain at its C-terminal end [16]. SHP2 is prevented from being active in typical conditions due to autoinhibition of the PTP domain by the N-SH2 domain. The N-SH2 domain binds to certain phosphotyrosine-containing peptides in response to growth factor or cytokine stimulation, resulting in a conformational shift that exposes the PTP domain and catalytic activation. Energy and specificity of the SHP2 binding to the C-SH2 domain are aided by this domain [17, 18].

SHP2 has been shown to promote activation of the RAS-mitogen-activated protein kinase (MAPK) pathway in response to a wide range of agonists and in a variety of cell types. This canonical signaling cascade plays a critical role in a variety of cellular processes, including migration, differentiation, survival, and proliferation [19]. SHP2 is found in a variety of human tissues, with the highest levels found in the heart, brain, and skeletal muscle [20, 21], which means that once the PTPN11 gene is mutated, it is likely to affect the normal development and function of these organs to some extent.

PTPN11 is known as the most important pathogenic gene for Noonan syndrome. Noonan syndrome is a genetic disorder characterized by CHDs, short stature, and facial dysmorphia or other malformations. About 80% of Noonan syndrome patients suffer from CHD, such as pulmonary valve stenosis and septal defect [22, 23]. In this study, we collected nine unrelated CHD families. Given that PTPN11 mutations were found in both Noonan syndrome and nonsyndromic patients and that the CHD phenotype was present in all patients, we hypothesize that PTPN11 gene mutations may also be the genetic risk factor for isolated CHD development.

## 2. Materials and Methods

### 2.1. Study Subjects

There were 681 CHD patients from the Children's Hospital of Fudan University, nine of whom came from nine unrelated families, as well as 399 unaffected healthy individuals who served as controls. All sporadic CHD were isolated CHD, excluding syndromes or extracardial malformations. Experiments were approved by the Ethics Committee of Children's Hospital of Fudan University and were conducted in compliance with the Helsinki Declaration. Informed consent was obtained from every patient.

### 2.2. Whole-Exome Sequencing and Sanger Sequencing

Genomic DNA samples from nine separate CHD families were subjected to whole-exome sequencing. We screened for unique or rare coding variants (absence or minor allele frequency (MAF) < 0.01% in gnomAD_exome_EAS) and predicted deleterious candidates (at least damaging predicted by SIFT, PolyPhen2, and MutationTaster prediction programs and combined annotation dependent depletion (CADD) score value > 20). Through the use of Sanger sequencing, the discovered candidate gene mutations were confirmed.

As stated in Table S1, the sequences of the forward and reverse primers were designed online using the NCBI Primer creating tool. PrimeSTAR® Max DNA Polymerase (Takara, Shiga, Japan) were used in the polymerase chain reaction (PCR). Shanghai Jie Li Biotechnology Co., Ltd (Shanghai, China) sequenced the PCR products. Mutation Surveyor Software was used to evaluate the sequence data.

### 2.3. Plasmids and Site-Directed Mutagenesis

The PTPN11-pcDNA 3.1-Flag plasmid was purchased from ShanghaiGeneray Biotech Company (Shanghai, China). Site-directed mutagenesis was performed to introduce eight variants—c.181G>A (p.D61N), c.188A>G (p.Y63C), c.218C>T (p.T73I), c.417G>C (p.E139D), c.574G>C (p.D192H), c.854T>C (p.F285S), c.922A>G (p.N308D), and c.1528C>G (p.Q510E)—into the PTPN11-pcDNA 3.1-Flag plasmid according to the instructions of the KOD-Plus-Mutagenesis Kit (Toyobo, Osaka, Japan). All plasmids were verified by DNA sequencing.

### 2.4. Cell Culture and Treatment

We used Dulbecco's modified Eagle medium supplemented with 10% FBS and 1% penicillin-streptomycin for the cultivation of HEK293T and Ac16 cells at 37°C with 5 percent CO_2_. Wild-type (WT) or mutant PTPN11 constructs were transfected into HEK293T or Ac16 cells using Lipofectamine 3000 reagent.

### 2.5. Transfection of Genes with Lentiviruses with SHP2 shRNA

To eliminate the disturbance of endogenous SHP2, we first designed and synthesized SHP2 shRNAs according to the Sigma website (https://www.sigmaaldrich.cn/CN/zh). SHP2 shRNA1 sequences were 5′-GGATTCAAATTCTAGTAATAG-3′; shRNA2, 5′-GCAGTTAAATTGTGCGCTGTA-3′; and shRNA3, 5′-TATACCCTTAACCAGTTTAAT-3′. Subcloned into a lentiviral vector, these oligonucleotides were then generated in HEK293T cells. Lentivirus suspension was added into the complete medium for gene transduction in HEK293T cells, which were divided into three groups: control, mock, and SHP2-RNAi (SHP2-shRNA1, 2, or 3 lentiviral vectors). Following transduction for 48 h, stable cell lines were selected with medium containing puromycin (2 *μ*g/mL) for 10 days.

### 2.6. Western Blotting

ERK1/2 phosphorylation experiments were carried out on transfected HEK293T cells that had been seeded in 6-well plates (70 percent to 80 percent confluence). Following transfection, cells were incubated for 48 h under serum-starved conditions and treated with 20 ng/mL epidermal growth factor (EGF) for 5 or 15 min or left unstimulated. Using a radioimmunoprecipitation technique, the total protein was recovered from the lysis buffer (Thermo Fisher Scientific, Waltham, MA, USA). Transfer membranes containing equal amounts of proteins were treated overnight at 4°C with specified primary antibodies and then at 37°C for two hours with secondary antibodies. The primary antibodies and dilutions were as follows: anti-SHP2 (1 : 3000, Santa Cruz Biotechnology, Dallas, TX, USA), anti-pERK1/2 (1 : 1000, Cell Signaling Technology, Danvers, MA, USA), and anti-Vinculin (1 : 5000, Abmart, Shanghai, China). Anti-rabbit and anti-mouse horseradish peroxidase- (HRP-) conjugated secondary antibodies were employed at 1 : 5000. Band density was quantified with ImageJ software.

### 2.7. Quantitative Reverse Transcription Polymerase Chain Reaction (qRT-PCR)

To measure the amount of total RNA, we used the TRIzol reagent (Invitrogen) to extract RNA from the various cells using NanoDrop 2000 (Thermo Fisher Scientific). The PrimeScript™ RT reagent Kit (Takara) was used to reverse transcribe 1 µg of total RNA into cDNA. qRT-PCR assays were carried out by the use of the TB Green Kit (Takara) on a QuantStudio 3 Real-Time PCR System (Thermo Fisher Scientific) as follows: denaturation at 95°C for 10 min, followed by 40 cycles at 95°C for 5 sec, 60°C for 40 sec, and 72°C for 45 sec. SHP2 primers were 5′-GGAGGAGAACGGTTTGATTCTT-3′ and 5′-CGAGTCGTGTTAAGGGGCTG-3′. *β*-Actin primers were 5′-CCTGGCACCCAGCACAAT-3′ and 5′-GGGCCGGACTCGTCATAC-3′, which was used as an internal control for standardization. The relative expression of genes was calculated and normalized using the delta-delta CT (2-*ΔΔ*Ct) method relative to *β*-actin. Independent experiments were done in triplicate.

### 2.8. Cell Proliferation Assay

The Cell Counting Kit-8 (CCK8) assays were used to detect cell proliferation. A cell density of 4,000 cells per well was used in a 96-well plate. The treated cells were then cultured for 24 h in an incubator with CO_2_ for complete adherence to the well. CCK8 solution (10 *μ*L) was added to each well at the given time points, and the cells were subsequently cultivated for four hours at 37°C. A microplate reader was used to measure the absorbance of each well at 450 nm. A curve was plotted based on the OD value. For the backdrop correction, only medium-filled wells were used. The experiment was repeated three times in each group.

### 2.9. Wound Healing Assay

A 6-well plate was injected with cells from each group, and they were allowed to grow overnight to create confluent monolayers. Each group's monolayer was scratched using a sterile 200 *μ*L pipette tip. Next, cells were rinsed three times with PBS to eliminate floating cells and then cultivated for 24 hours in DMEM with 0% FBS. At 0 h, 12 h, and 24 h, the wounds were photographed using an inverted microscope. Analysis of the wound region was carried out using ImageJ.

### 2.10. Statistical Analysis

GraphPad Prism software (version 8.0, GraphPad Inc., San Diego, CA, USA) was used for statistical analysis and graph creation. All data were presented as the mean ± standard error of mean based on at least three separate studies. A one-way analysis of variance or Student's *t*-test was used, depending on the situation, to assess whether the results were significant. Two-side *p* < 0.05 was considered statistically significant.

## 3. Results

### 3.1. Identification of PTPN11 Variants in CHD Families

In this study, we first performed whole-exome sequencing on nine probands from nine unrelated CHD families to identify rare pathogenic coding variants underlying the CHD development, and the clinical phenotype of each proband in these families is listed in Table S2. By stringently filtering, we identified a total of eight novel or rare deleterious heterozygous missense variants in PTPN11 gene, which were present in these nine individual probands, including c.181G>A (p.D61N), c.188A>G (p.Y63C), c.218C>T (p.T73I), c.417G>C (p.E139D), c.574G>C (p.D192H), c.854T>C (p.F285S), c.922A>G (p.N308D), and c.1528C>G (p.Q510E). Sanger sequencing of these probands and their unaffected family members confirmed that six damaging variants were de novo in seven CHD families, and two variants in two other CHD families were inherited from their unaffected parents, indicating its incomplete penetrance (Figures 1(a) and 1(b)).

The PTPN11 c.181G>A (p.D61N) mutation was recurrent in two probands from family 1 and family 2. The proband in family 1 was a 3-year-old male with atrial septal defect (ASD) and persistent left superior vena cava. The other affected individual in family 2 was a 7-year-old female presenting only with ASD. This variant is de novo novel (absent in gnomAD_genome_EAS) in the two families and predicted to be deleterious (CADD = 32, SIFT = D, Polyphen2 = D). The mutation substitutes the evolutionarily conserved residue in the N-SH domain of PTPN11.

The proband in family 3 was a 3-year-old male with pulmonary stenosis (PS) and patent foramen ovale (PFO) and carried a PTPN11 c.188A>G (p.Y63C) variant which was exceedingly rare (MAF = 5.43656*E* − 05 in gnomAD_genome_EAS) and predicted to be deleterious (CADD = 28.1, SIFT = D, Polyphen2 = D), involving acid amino Tyr-to-Cys substitution at position 63. However, this variant was confirmed to be inherited from his unaffected mother, reflecting its incomplete penetrance.

The proband in family 4 was a 1-year-old male infant, who was diagnosed with ASD and PS and accompanied by craniofacial dysmorphism, cryptorchidism, and auditory abnormality, a typical characteristic of Noonan syndrome. The PTPN11 c.218C>T (p.T73I) mutation observed in this family was a missense variant and predicted to be damaging (CADD = 27.4, SIFT = D, Polyphen2 = D). The variant was absent in his normal parents and other family members and confirmed to be de novo.

The PTPN11 c.417G>C (p.E139D) variant was discovered in proband 5 in family 5, a 2-year-old male suffering from ASD, PFO, and patent ductus arteriosus (PDA), as well as craniofacial dysmorphism and chest deformity, a Noonan syndrome. The variant, which was absent in the public database, was confirmed as a de novo missense mutation predicted to be highly deleterious (CADD = 25, SIFT = D, Polyphen2 = D).

The proband in family 6 was a 1-year-old male who presented with ASD, VSD, PDA, and aortic coarctation. The PTPN11 c.574G>C (p.D192H) was absent in the public database and unreported previously, which was predicted to be damaging (CADD = 24.8, SIFT = D, Polyphen2 = B). The p.D192H was inherited from the proband's healthy mother, showing its incomplete penetrance in this case.

The PTPN11 c.854T>C (p.F285S) variant was identified in proband 7 who was a 3-year-old female. She was diagnosed with ASD, PS, PFO, and stenosis of the right ventricular outflow tract. The p.F285S variant was identified as a novel missense mutation which is highly deleterious (CADD = 32, SIFT = D, Polyphen2 = D), which was confirmed to be de novo in this family.

The proband in family 8 was a 10-year-old male with PFO, who carried a PTPN11 c.922A>G (p.N308D) variant, which was a rare missense variant showing high deleteriousness (CADD = 23.6, SIFT = D, Polyphen2 = B) and validated to be de novo.

The PTPN11 c.1528C>G (p.Q510E) variant was present in proband 9 in family 9 who was a 2-year-old male patient and presented with ASD, PFO, PDA, and hypertrophic cardiomyopathy. The observed variant p.Q510E was a missense type and show highly damaging by multiple predicted software (CADD = 26.5, SIFT = D, Polyphen2 = D). Sanger sequencing of the proband and his unaffected parents confirmed this variant as de novo.

All of the abovementioned variations in the PTPN11 gene altered evolutionarily conserved amino acids, and they were all found in important functional domains of the protein (Figure 2(a)2(b) and 2(c)). Moreover, among these nine CHD families, seven of them showed de novo PTPN11 mutations, and two families harbored PTPN11 mutations inherited from their unaffected parents, indicating its incomplete penetrance. Although PTPN11 gene is known as the pathogenic gene of Noonan syndrome, in our study cohort of nine families, only probands 4 and 5 presented three main characteristics of Noonan syndrome. Based on the fact that all patients suffered from CHD regardless of whether they had Noonan syndrome, we concluded that PTPN11 mutations may also be the main genetic factor for CHD.

### 3.2. Association of Damaging PTPN11 Variants with the Risk of CHD Development

To further investigate the prevalence of PTPN11 variants and its association with the risk of CHD, we then carried out targeted exon sequencing of PTPN11 gene in additional 672 individuals with CHD and 399 unrelated healthy controls.

Eight additional CHD probands harbored seven novel or rare heterozygous missense PTPN11 variants that fulfilled filtering criteria (absent in gnomAD_genome_EAS or MAF < 0.1%, CADD > 20). The identified PTPN11 mutation information is shown in Table S3.

In total, among sporadic cases of CHD, 8 of 672 (1.19%) had a PTPN11 variant that passed a priori filtering constraints. Fisher's exact test reveals a significant association of PTPN11 variations with the risk of CHD development (Fisher's exact test, *P* = 0.0289).

### 3.3. The Distribution of Different Subtypes in CHD Patients with PTPN11 Variants

We then further observed the distribution of different subtypes in CHD patients with PTPN11 mutations. A total of 17 CHD patients harbored 15 novel or rare heterozygous missense variants in PTPN11 gene. Table S4 shows the distribution of CHD subtypes in familial and sporadic cases. Of the 9 patients from the family, 7 show the highest incidence of ASD (77.8%). Among the 8 patients from sporadic CHD cases, 3 subjects presented with a higher prevalence of ASD phenotype (37.5%). Together, among the 17 patients with PTPN11 variants, ASD was the main CHD phenotype (58.8%, 10/17), indicating that ASD is a prominent phenotype in CHD patients with PTPN11 mutation.

### 3.4. PTPN11 Variants Alter RAS-MAPK Signaling Activity

SHP2 shRNA was used to knock down the expression of SHP2 in HEK293T cells, which was accomplished by the use of lentiviruses. We detected SHP2 levels with qRT-PCR or western blotting to validate knockdown efficiency. Compared to the shControl groups, levels of SHP2 mRNA in the SHP2 shRNA1, 2, and 3 subgroups were reduced by 81.37%, 79.93%, and 73.58%, respectively (Figure 3(a)). Western blot assays demonstrated that SHP2 levels in these three subgroups were significantly reduced by 77.74%, 78.61%, and 71.49%, respectively (Figure 3(b)).

The RAS-MAPK pathway plays an important role during weeks 2-8 of embryonic development, which is the most critical cardiac development period. ERK1/2 is a key protein in this pathway, and its phosphorylation level can reflect RAS-MAPK signaling activity. To clarify the effect of PTPN11 mutations on RAS-MAPK signaling, we overexpressed WT and mutant PTPN11 in shRNA knockdown HEK293T cells. Following transfection, cells were serum-starved and treated with 20 ng/mL EGF for 5 or 15 min or left unstimulated. Cells were then collected and lysed for immunoblotting. We determined the effects of PTPN11 mutations on ERK1/2 phosphorylation. As shown in Figures 4(a) and 4(b), at the 5 min time point, pERK1/2 was significantly increased for the SHP2-D61N, SHP2-Y63C, SHP2-T73I, SHP2-D192H, SHP2-F285S, and SHP2-N308D mutations by 41.13%, 20.40%, 63.26%, 89.85%, 31.36%, and 86.57%, respectively, while it was significantly reduced for the SHP2-Q510E mutation by 20.36%. After 15 min, the pERK1/2 of the abovementioned mutation groups had the same increased or decreased trends, but there was no statistical difference except for SHP2-Y63C and SHP2-Q510E. ERK1/2 phosphorylation levels were not significantly different between cells producing SHP2-E139D mutants and the WT protein in this study. These results suggested that upon EGF stimulation, PTPN11 mutations can promote or inhibit the activation of the RAS-MAPK signaling pathway to different degrees.

### 3.5. SHP2 Mutations Promote Ac16 Cell Proliferation

The effect of SHP2 mutations on Ac16 cell proliferation ability was determined with CCK8 assays. Compared with the WT group, the absorbances of the SHP2-E139D, SHP2-D192H, SHP2-F285S, SHP2-N308D, and SHP2-Q510E mutant groups increased by 10.50%, 8.43%, 13.20%, 20.36%, and 18.73% after 72 h, respectively, and all of these increases were statistically significant (Figure 5). Thus, the data indicated that SHP2 mutations enhanced Ac16 cell proliferation.

### 3.6. SHP2 Mutations Enhance Ac16 Cell Migration

We performed wound healing assays to examine the influences of PTPN11 gene mutations on cell migration. Images were taken 0, 12, and 24 h after the scratch to record the size of the scratched areas to reflect cellular migration ability. Compared with the WT group, SHP2-D192H, SHP2-F285S, SHP2-N308D, and SHP2-Q510E mutant groups had increased cell migration by 57.43%, 45.96%, 46.48%, and 50.28% after 12 h and by 48.34%, 34.71%, 32.00%, and 35.56% after 24 h, respectively (Figures 6(a) and 6(b)). The differences were statistically significant at 24 h, demonstrating that Ac16 cell migration was increased by SHP2-D192H, SHP2-F285S, SHP2-N308D, and SHP2-Q510E expression.

## 4. Discussion

In this study, we performed whole-exome sequencing on nine unrelated CHD nuclear families and identified eight rare deleterious missense variants of PTPN11 gene in nine probands by stringently filtering criteria. In seven CHD families, six of these variations were found to be de novo, confirming their pathogenicity. Moreover, two variants in two CHD families were inherited from their unaffected parents, indicating its incomplete penetrance. To further assess the association of the PTPN11 variants with the risk of CHD development, we carried out targeted sequencing to analyze the PTPN11 exon variants in 672 sporadic CHD cases and 399 unrelated controls.

Among the sporadic patients, we compared the prevalence of PTPN11 variants in CHD patients and controls and observed a significant association of PTPN11 variations with CHD development (*P* = 0.0289).

PTPN11 gene mutations are one of the main causes of Noonan syndrome which is characterized by distinctive facial features, short stature, chest deformity, and other comorbidities. In addition to these features, about 80% of patients also have CHD, including pulmonary stenosis, hypertrophic cardiomyopathy, and atrial or ventricular septal defects [24]. In isolated CHD, many of the same genes that play a key role in syndromic CHD can also be found to be implicated, such as NOTCH1 (Adams-Oliver syndrome) [25], TBX5 (Holt-Oram syndrome) [26], and JAG1 (Alagille syndrome) [27]. We may be able to identify some of the genetic causes of isolated CHD by studying the genetic foundation of syndromic CHD [28].

It is well known that the CHD phenotype among individuals with PTPN11 mutations differ from those with Noonan syndrome and LEOPARD syndrome, in that pulmonary stenosis is most common in Noonan syndrome [29, 30], whereas hypertrophic cardiomyopathy prevails in LEOPARD syndrome [31]. However, in our study, the ASD subphenotype was most prominent in CHD patients with PTPN11 mutations. This observation of phenotypic discrepancies in CHD may be explained by the following three aspects: first, the cases we collected focused on CHD rather than syndromes caused by PTPN11 mutations; second, the CHD phenotype may vary in different regions and races/ethnicities; and third, nongenetic factors, such as genetic heterogeneity, varied penetrance, a wide range of expressivity, and other influences, may have an impact on phenotypic development [28, 32]. Two 2019 studies of PTPN11 gene abnormalities based on the Chinese population also support our observations [23, 33]. The collective evidence showed that ASD was a prominent CHD phenotype in patients with PTPN11 variants in the Chinese population.

For the eight PTPN11 gene mutations found in the families, we conducted structural and functional analysis. A number of amino acid substitutions affect evolutionarily conserved residues, all of which are found in critical regions of the protein, suggesting that they were likely to affect domain function and protein conformation, leading to gene abnormalities. Both the pathogenicity website predictions and the gnomAD data suggested that they were pathogenic mutations, which are probably related to the pathogenesis of CHD.

The RAS-MAPK signaling pathway is a typical signal cascade that exists in most cells; it transduces extracellular signals such as growth factors and hormones into the cells to promote cell proliferation, differentiation, metabolism, and many other important cell activities. The embryonic timing of 2-8 weeks is the most critical period for heart development, and RAS-MAPK signaling plays an important role. Perturbation of this pathway is likely to cause heart development defects. SHP2 acts as a phosphatase in the RAS-MAPK signaling pathway. Once stimulated, it activates RAS by binding to the interacting protein and then induces the RAF-MEK-ERK signaling cascade through a series of phosphorylation reactions. Finally, ERK enters the nucleus to regulate gene transcription, allowing the cell to respond to stimulus signals [19].

As a necessary member to maintain the activation of the RAS-MAPK signaling pathway [34], SHP2 may interfere with the RAS-MAPK signaling pathway to affect basic cellular activities, leading to CHD pathogenesis. In 2019, Yang et al. found that the phosphorylation level of ERK1/2 after SHP2-E76K transduction was significantly higher than after SHP2-WT transduction or that in the control group. Moreover, SHP2-E76K promoted cell proliferation and migration ability, which were greatly inhibited by the ERK inhibitor U0126, suggesting that SHP2-E76K promotes cell proliferation and migration partially by relying on ERK [35].

Proper formation of the cardiac structure requires normal cellular processes such as proliferation and migration. Nakamura et al. found that SHP2-deficient neural crest cells failed to migrate into the developing outflow tract in the developing heart, and the embryos displayed persistent truncus arteriosus and abnormalities of the great vessels [6]. Krenz et al. showed that in cells produced from endothelial stem cells, overexpression of SHP2-Q79R led to enhanced cell proliferation and decreased apoptosis in the cushion mesenchyme and endothelium, resulting in larger endocardial cushions [14]. In addition, abnormal cellular processes, such as proliferation and migration, may not only directly affect the maturation of the heart structure but also affect the blood flow distribution of the developing heart, leading to secondary cardiovascular defects [36].

Accumulating evidence indicated that mutations of PTPN11 gene have been linked to a wide range of cardiac abnormalities, underscoring the need for fine-tuning phosphorylation processes during heart embryo development [19, 37]. Here, we showed that increased or decreased activity in RAS-MAPK signaling caused by abnormal PTPN11 can promote cell proliferation and migration, reflecting that a precise level or duration of RAS-MAPK activity was required during heart development to elicit a specific proliferative or migration response.

SHP2's ubiquitous expression and its pivotal functions in cell activities endow PTPN11 with key functions during embryonic development. Beyond the RAS-MAPK signaling pathway, SHP2 also plays important roles in phosphoinositide 3-kinase-AKT, Janus kinase-signal transducer and activator of transcription, nuclear factor-*κ*B, RHO, and nuclear factor of activated T-cell signaling pathways, implying that the disease may be caused by concomitant dysregulation of multiple pathways [37, 38]. Besides, biochemical and cell biological analyses and experiments with small molecule compounds have demonstrated that SHP2 has both phosphatase-dependent and phosphatase-independent functions [39]. In the future, it is necessary to combine stem cell models, animal models, and other advanced technologies to further explore the pathogenic mechanism of SHP2.

## 5. Conclusion

We found 15 heterozygous missense mutations in the PTPN11 gene in 17 patients from 9 families and 672 sporadic cases, and these novel and rare mutations expanded the spectrum of pathogenic genetic mutations in the PTPN11 gene. Among them, mutations in 7 out of 9 families were de novo, adding to the evidence for pathogenicity. ASD was a prominent phenotype in CHD associated with PTPN11 gene mutation. The changes in signaling pathway activity and cell proliferation and migration due to PTPN11 mutations all supported the putative pathogenicity of these variants in CHD. Our findings reveal that the PTPN11 variants are associated with an increased risk of CHD development and can be considered an important susceptible genetic event for CHD, especially the ASD subphenotype.

## Figures and Tables

**Figure 1:** Affected families' PTPN11 variations were identified. (a) Pedigrees were shown for the 9 families. The arrows represent the probands, and black circles or squares represent the affected individuals. (b) Sanger sequencing confirmation.

**Figure 2:** Locations and conservation of PTPN11 mutations. (a) The positions of all mutations are indicated in the genomic structure of PTPN11. (b) Schematic representation of the structure of the SHP2 protein and positions of the residues affected by the identified PTPN11 mutations. (c) The residues are conserved from human to zebrafish (prepared from the UCSC genome browser).

**Figure 3:** Efficient knockdown of SHP2 by shRNA lentivirus confirmed by qRT-PCR and immunoblotting. (a) SHP2 mRNA levels in the cell lines. (b) Quantitative study of SHP2 expression using western blots (^∗∗∗^*p* < 0.001,  ^∗∗∗∗^*p* < 0.0001). Experiments were repeated three times with three replicates in each experiment.

**Figure 4:** The effect of PTPN11 variants on ERK1/2 phosphorylation. (a) pERK1/2 was analyzed by transiently expressing the WT and mutant constructs in shRNA knockdown HEK293T cells. Expression of the SHP2-D61N, SHP2-Y63C, SHP2-T73I, SHP2-D192H, SHP2-F285S, and SHP2-N308D mutants resulted in increased ERK1/2 phosphorylation compared with cells expressing WT proteins, and SHP2-Q510E mutation decreased phosphorylation. (b) Quantification of the immunoblot results. ^∗^*p* < 0.05. Experiments were repeated three times with three replicates in each experiment.

**Figure 5:** CCK8 assays showed that SHP2 mutations promoted Ac16 cell proliferation (^∗^*p* < 0.05). Experiments were repeated three times with three replicates in each experiment.

**Figure 6:** SHP2 enhanced Ac16 cell migration. (a) Representative images of wound areas immediately after scratching (top), after 12 h (middle), and after 24 h (bottom) by SHP2-D192H, SHP2-F285S, SHP2-N308D, and SHP2-Q510E. (b) Quantification of wound areas after 24 h. ^∗^*p* < 0.05,  ^∗∗^*p* < 0.01. Experiments were repeated three times with three replicates in each experiment.

## Data Availability

The data that support the findings of this study are available from the corresponding authors upon reasonable request.

## Supplementary Materials

Supplementary 1 Table S1: Sanger sequencing primer pair for detecting PTPN11 mutations.

Supplementary 2 Table S2: clinical characteristics in CHD patients with PTPN11 mutations.

Supplementary 3 Table S3: PTPN11 variants detected in both pedigrees and sporadic cases.

Supplementary 4 Table S4: cardiac phenotypes observed in pedigrees and sporadic cases.

## References

[1] Zhao Q. M., Liu F., Wu L., Ma X. J., Niu C., Huang G. Y. (2019). Prevalence of congenital heart disease at live birth in China. *The Journal of Pediatrics*.

[2] Shabana N. A., Shahid S. U., Irfan U. (2020). Genetic contribution to congenital heart disease (CHD). *Pediatric Cardiology*.

[3] Williams K., Carson J., Lo C. (2019). Genetics of congenital heart disease. *Biomolecules*.

[4] Blue G. M., Kirk E. P., Giannoulatou E. (2017). Advances in the genetics of congenital heart disease: a clinician's guide. *Journal of the American College of Cardiology*.

[5] Nakamura T., Colbert M., Krenz M. (2007). Mediating ERK 1/2 signaling rescues congenital heart defects in a mouse model of Noonan syndrome. *The Journal of Clinical Investigation*.

[6] Nakamura T., Gulick J., Colbert M. C., Robbins J. (2009). Protein tyrosine phosphatase activity in the neural crest is essential for normal heart and skull development. *Proceedings of the National Academy of Sciences of the United States of America*.

[7] Araki T., Mohi M. G., Ismat F. A. (2004). Mouse model of Noonan syndrome reveals cell type- and gene dosage-dependent effects of Ptpn11 mutation. *Nature Medicine*.

[8] Jopling C., van Geemen D., den Hertog J. (2007). Shp2 knockdown and Noonan/LEOPARD mutant Shp2-induced gastrulation defects. *PLoS Genetics*.

[9] Bonetti M., Paardekooper Overman J., Tessadori F., Noël E., Bakkers J., den Hertog J. (2014). Noonan and LEOPARD syndrome Shp2 variants induce heart displacement defects in zebrafish. *Development*.

[10] Miura K., Wakayama Y., Tanino M. (2013). Involvement of EphA2-mediated tyrosine phosphorylation of Shp2 in Shp2-regulated activation of extracellular signal-regulated kinase. *Oncogene*.

[11] Langdon Y. G., Goetz S. C., Berg A. E., Swanik J. T., Conlon F. L. (2007). SHP-2 is required for the maintenance of cardiac progenitors. *Development*.

[12] Langdon Y., Tandon P., Paden E., Duddy J., Taylor J. M., Conlon F. L. (2012). SHP-2 acts via ROCK to regulate the cardiac actin cytoskeleton. *Development*.

[13] Araki T., Chan G., Newbigging S., Morikawa L., Bronson R. T., Neel B. G. (2009). Noonan syndrome cardiac defects are caused by PTPN11 acting in endocardium to enhance endocardial-mesenchymal transformation. *Proceedings of the National Academy of Sciences of the United States of America*.

[14] Krenz M., Gulick J., Osinska H. E., Colbert M. C., Molkentin J. D., Robbins J. (2008). Role of ERK1/2 signaling in congenital valve malformations in Noonan syndrome. *Proceedings of the National Academy of Sciences of the United States of America*.

[15] Chen B., Bronson R. T., Klaman L. D. (2000). Mice mutant for Egfr and Shp2 have defective cardiac semilunar valvulogenesis. *Nature Genetics*.

[16] Neel B. G., Gu H., Pao L. (2003). The 'Shp'ing news: SH2 domain-containing tyrosine phosphatases in cell signaling. *Trends in Biochemical Sciences*.

[17] Hof P., Pluskey S., Dhe-Paganon S., Eck M. J., Shoelson S. E. (1998). Crystal structure of the tyrosine phosphatase SHP-2. *Cell*.

[18] Barford D., Neel B. G. (1998). Revealing mechanisms for SH2 domain mediated regulation of the protein tyrosine phosphatase SHP-2. *Structure*.

[19] Tajan M., de Rocca Serra A., Valet P., Edouard T., Yart A. (2015). SHP2 sails from physiology to pathology. *European Journal of Medical Genetics*.

[20] Ahmad S., Banville D., Zhao Z., Fischer E. H., Shen S. H. (1993). A widely expressed human protein-tyrosine phosphatase containing src homology 2 domains. *Proceedings of the National Academy of Sciences of the United States of America*.

[21] Bastien L., Ramachandran C., Liu S., Adam M. (1993). Cloning, expression and mutational analysis of SH-PTP2, human protein-tyrosine phosphatase. *Biochemical and Biophysical Research Communications*.

[22] Athota J. P., Bhat M., Nampoothiri S. (2020). Molecular and clinical studies in 107 Noonan syndrome affected individuals with PTPN11 mutations. *BMC Medical Genetics*.

[23] Li X., Yao R., Tan X. (2019). Molecular and phenotypic spectrum of Noonan syndrome in Chinese patients. *Clinical Genetics*.

[24] Romano A. A., Allanson J. E., Dahlgren J. (2010). Noonan syndrome: clinical features, diagnosis, and management guidelines. *Pediatrics*.

[25] Page D. J., Miossec M. J., Williams S. G. (2019). Whole exome sequencing reveals the major genetic contributors to nonsyndromic Tetralogy of Fallot. *Circulation Research*.

[26] Smemo S., Campos L. C., Moskowitz I. P., Krieger J. E., Pereira A. C., Nobrega M. A. (2012). Regulatory variation in a TBX5 enhancer leads to isolated congenital heart disease. *Human Molecular Genetics*.

[27] Bauer R. C., Laney A. O., Smith R. (2010). Jagged1 (JAG1) mutations in patients with tetralogy of Fallot or pulmonic stenosis. *Human Mutation*.

[28] Nees S. N., Chung W. K. (2020). The genetics of isolated congenital heart disease. *American Journal of Medical Genetics. Part C, Seminars in Medical Genetics*.

[29] Linglart L., Gelb B. D. (2020). Congenital heart defects in Noonan syndrome: diagnosis, management, and treatment. *American Journal of Medical Genetics. Part C, Seminars in Medical Genetics*.

[30] Tartaglia M., Kalidas K., Shaw A. (2002). PTPN11 mutations in Noonan syndrome: molecular spectrum, genotype-phenotype correlation, and phenotypic heterogeneity. *American Journal of Human Genetics*.

[31] Limongelli G., Pacileo G., Marino B. (2007). Prevalence and clinical significance of cardiovascular abnormalities in patients with the LEOPARD syndrome. *The American Journal of Cardiology*.

[32] Lee C. L., Tan L. T. H., Lin H. Y. (2020). Cardiac manifestations and gene mutations of patients with RASopathies in Taiwan. *American Journal of Medical Genetics. Part A*.

[33] Chen H., Li X., Liu X. (2019). Clinical and mutation profile of pediatric patients with RASopathy-associated hypertrophic cardiomyopathy: results from a Chinese cohort. *Orphanet Journal of Rare Diseases*.

[34] Yu Z. H., Xu J., Walls C. D. (2013). Structural and mechanistic insights into LEOPARD syndrome-associated SHP2 mutations∗. *The Journal of Biological Chemistry*.

[35] Yang F., Xu M., Wang S. (2019). Gain-of-function E76K-mutant SHP2 promotes cell proliferation, metastasis, and tumor growth in glioblastoma through activation of the ERK/CREB pathway. *OncoTargets and therapy*.

[36] Krenz M., Yutzey K. E., Robbins J. (2005). Noonan syndrome mutation Q79R in Shp2 increases proliferation of valve primordia mesenchymal cells via extracellular signal-regulated kinase 1/2 signaling. *Circulation Research*.

[37] Lauriol J., Jaffré F., Kontaridis M. I. (2015). The role of the protein tyrosine phosphatase SHP2 in cardiac development and disease. *Seminars in Cell & Developmental Biology*.

[38] Mohi M. G., Neel B. G. (2007). The role of Shp2 ( PTPN11 ) in cancer. *Current Opinion in Genetics & Development*.

[39] Guo W., Xu Q. (2020). Phosphatase-independent functions of SHP2 and its regulation by small molecule compounds. *Journal of Pharmacological Sciences*.

